# Application of Emergency Specialist Nursing Combined with Green Channel Mode in Patients with Limb Amputation

**DOI:** 10.1155/2022/3838928

**Published:** 2022-04-19

**Authors:** Zaiyun Qian, Min Wang, Tonglong Xu

**Affiliations:** Wuxi 9th People's Hospital Affiliated to Soochow University, Liangxi Road, No. 999, Binhu District, Wuxi, Jiangsu, China

## Abstract

**Background:**

The treatment of limb amputation is always a challenge to emergency medical staff. The success of replantation of severed limbs requires not only emergency professional nursing measures but also rapid transport against time. We that found emergency specialist nursing combined with green channel mode can effectively improve the success rate of amputated limb replantation surgery.

**Methods:**

From September 2017 to August 2020, the medical records of 80 patients with severed limb replantation treated by the emergency department of our hospital were collected and divided into the control group and the experimental group. 36 patients in the control group were emergency patients treated from September 2017 to May 2019. These patients did not take appropriate emergency specialist nursing measures and opened green channels at that time; the other 44 patients were in the experimental group, for emergency patients treated from June 2019 to August 2020. These patients have received emergency specialist care and opened a green channel. We recorded the gender, age, preoperative examination time, and success rate of amputated limb replantation surgery of the two groups of patients.

**Results:**

The age of the patients in the control group was 41.17 ± 8.00 years old, and the age of the patients in the experimental group was 41.07 ± 7.31 years old (*P* > 0.05). The preoperative examination time of the patients in the control group was 46.53 ± 4.11 min, and the preoperative examination time of the patients in the experimental group was 40.34 ± 5.85 min (*P* < 0.05); the replantation success rate of the control group was 72.2%, and the replantation success rate of the experimental group was 81.8% (*P* < 0.05).

**Conclusion:**

Standardized emergency specialist nursing measures combined with green channel mode can effectively shorten the preoperative examination time and help improve the success rate of amputated limb replantation surgery.

## 1. Introduction

With the development of urban and industrial mechanization, the incidence of serious trauma caused by traffic accidents and mechanical equipment is increasing significantly, and limb amputation injuries caused by such high-energy injuries are more and more common. Emergency care of such severe trauma has always been a challenge for our emergency department. The trauma treatment center of our hospital has been undertaking the first aid work for patients with severe trauma in this city and nearby areas. Such patients often have a hemorrhagic shock when they are sent to the hospital, which seriously affects the prognosis of the patients and even threatens their lives.

Proximal limb amputations caused severe functional and psychological consequences to patients, which might also lead to significant disturbances in quality of life. The lower limb amputation might cause loss operation, and regaining functional mobility, developing independence, and improving quality of life are significant [1]. Rapid medical response teams and poor public awareness about the procedure are important for the prognosis of these patients. Upper extremity amputations are connected with morbidity. After the success of limb replantation, there have been many replantations of digits, hands, and limbs around the world [1].

This article retrospectively studied 80 cases of amputated limb replantation treated in the emergency department of our hospital and found that standardized emergency specialist nursing measures combined with green channel mode [2] can effectively improve the success rate of amputated limb replantation surgery.

## 2. Materials and Methods

### 2.1. General Materials

Inclusion criteria are as follows: (1) unilateral limb amputation injury, (2) normally healthy and no other diseases, (3) 18-50 years old, and (4) no history of trauma to the injured limb.

Exclusion criteria are as follows: (1) combined with other injuries, (2) multisegment limb amputation, and (3) have been treated in other hospitals.

From September 2017 to August 2020, according to the inclusion and exclusion criteria, the medical records of 80 patients with severed limb replantation treated by the emergency department of our hospital were collected and divided into the control group and the experimental group. 36 patients in the control group were emergency patients treated from September 2017 to May 2019. These patients did not take appropriate emergency specialist nursing measures and opened green channels at that time; the other 44 patients were in the experimental group, for emergency patients treated from June 2019 to August 2020. These patients have received emergency specialist care and opened a green channel. We recorded the gender, age, preoperative examination time, and the success rate of amputated limb replantation surgery of the two groups of patients. Written notifications signed by patients were added in clinical research methods.

### 2.2. Emergency Specialist Nursing Measures

#### 2.2.1. Open the Green Channel

The emergency triage desk will immediately escort the patient to the emergency room after accepting the patient, and at the same time notify the medical staff to arrive at the scene, prepare rescue equipment and medicines, and urgently coordinate the emergency laboratory, imaging department, operating room, and other related departments to accept patients. Arrange the escort to accompany the patient throughout the whole process until the patient is sent to the operating room, and the patient will be treated first and then paid, so as to shorten the time from admission to the operating room for surgical treatment, to achieve zero waiting for treatment.

#### 2.2.2. Rapid Identification of Shock

Patients with severed limb injury often bleed a lot. The systemic small vessels constrict and spasm during the compensatory stage of shock, and blood flow is mainly returned through direct access or arteriovenous short-circuit. The blood pressure during this stage is often normal or slightly lower than normal or even slightly increased, but the pulse pressure difference is low. During the compensatory stage of shock, tissue perfusion and oxygenation are significantly reduced and manifested as a drop in the blood oxygen saturation. We calculated the shock index, quickly identified whether the patient was in shock, and immediately performed antishock treatment.

#### 2.2.3. Antishock Treatment

(1) Give the patient a supine shock position, keep the airway unobstructed, monitor the vital signs continuously, and detect and record the changes in time. Raise the room temperature and use a thermostatic quilt cover to keep warm to prevent hypothermia. (2) Quickly establish venous access to supplement blood volume. Select the thick veins in the elbow and neck, quickly establish two venous channels with an indwelling needle, and inject 500 ml of balanced solution intravenously, respectively. (3) The stump of the amputated limb is compressed with a sterile dressing and then fixed with a roll-type splint. Use elastic bandages as pads to tie a pneumatic tourniquet at the proximal 1/3 of the upper arm or thigh. Apply sufficient pressure to the proximal part of the traumatic limb to block arterial and venous blood flow to achieve hemostasis.

#### 2.2.4. Preservation of Amputated Limbs

Put the amputated limb into a special insulation box with a lid (Figure 1), put the amputated limb into a disposable sterile fresh-keeping bag, and place an ice pack around the fresh-keeping bag to keep the temperature at about 4°C. Place a label on the outside of the fresh-keeping bag of the severed limb, indicating the injured person's name, age, location, and time of injury.

#### 2.2.5. Actively Make Preoperative Preparations

X-ray and CT examinations are routinely performed at the amputated limb, and other suspicious parts also need to be examined to confirm the diagnosis. Complete the blood tests and follow up the test results in time. During the rescue, make preoperative preparations, such as skin preparation, drug allergy testing, and indwelling catheterization, timely notify the relevant departments for consultation, and prepare for the operation in the shortest time.

#### 2.2.6. Analgesia and Psychological Care

Correctly assess the degree, location, time, and cause of the patient's pain, and take corresponding pain relief measures, such as properly raising the affected limb and instructing the patient to breathe deeply. In the case of severe pain, report to the doctor to use effective analgesic drugs as prescribed by the doctor and make a record. Pay attention to listening to the main complaints of the patients, explain the specific conditions of the disease to the patients, tell the successful cases of the operation to enhance the confidence of the patients, gain the trust of the patients with cordial services, and improve the compliance of the patients.

### 2.3. Data Processing and Statistical Analysis

Use SPSS 23.0 statistical software package (SPSS Inc., Chicago, IL) for statistical analysis. Data are expressed as mean ± standard deviation. Data are compared by an independent sample *t*-test. *P* < 0.05 indicates that the difference is statistically significant.

## 3. Results

This study collected the information of patients and compared the age of two groups. The age of the patients in the control group was 41.17 ± 8.00 years old, while the age of the patients in the experimental group was 41.07 ± 7.31 years old, which has no significant difference (*P* > 0.05). Then, we compared the preoperative examination time of the patients. The preoperative examination time in the control group was 46.53 ± 4.11 min, which is significantly longer than that in the experimental group (40.34 ± 5.85 min, *P* < 0.05). The replantation success rate of the control group was 72.2%, and the replantation success rate of the experimental group was 81.8%, which also has significant difference (*P* < 0.05) (Table 1).

## 4. Discussion

In our study, the preoperative examination time of the patients in the experimental group was significantly lower than that of the control group, and the success rate of the amputated limb replantation in the experimental group was significantly higher than that in the control group. After the amputated patient is admitted to the hospital, we first evaluate the patient's general condition and the condition of limb replantation. If the damage is extremely serious, we can only treat it with amputation [3]. Limb salvage surgery is time-limited (6-8 hours is the prime time), and how to get patients to the operating room as soon as possible is also a huge challenge for emergency medical staff. As the largest surgical center for replantation of amputated limbs in the surrounding area, our hospital has formed a mature rapid transport model. Rapid pre-examination and triage, timely opening of green channels, close connection of relevant examination departments, special personnel escort and transport, etc. all ensure that patients can complete preoperative examinations as quickly as possible.

In my country, amputation injuries caused by war and high-voltage electricity are relatively rare [4–6], mainly caused by traffic accidents. Such direct violent injuries often leave patients with some opportunities to save their limbs. Such patients are often accompanied by massive bleeding, but their blood pressure does not drop significantly during the compensatory stage of shock, which requires us to quickly identify the compensatory stage of shock. At this stage, the systemic small blood vessels constrict and spasm, and the blood flow mainly returns through direct access or arteriovenous short-circuit. The blood pressure is often normal or slightly lower than normal or even slightly increased, but the pulse pressure difference is reduced. At this stage, tissue perfusion and oxygenation will be significantly reduced, manifested as a drop in blood oxygen saturation. Therefore, we can quickly identify the compensatory stage of shock by pulse pressure difference and oxygen saturation and perform immediate infusion therapy. Restrictive fluid resuscitation can effectively control the blood pressure level of patients by strictly controlling the rate and amount of fluid infusion, which can not only improve the blood perfusion of important organs of the body but also stabilize the body's internal environment, thus reducing the incidence of complications. Of course, it is often controversial whether or not to save the limb [7–8]. When the patient's limb condition or general condition is extremely poor, we can only choose amputation [9–16]. However, Polcz [17] proposed that temporary use of endovascular shunt anastomosis can effectively improve the success rate of replantation.

For the treatment of the stump of the affected limb, we use a sterile dressing for compression dressing and then fix it with a roll-type splint. The splint is a new type of fracture fixation device made of IXPE (polyethylene cross-linked foamed plastic) wrapped with an aluminum plate. This type of splint can be freely shared and used together with bandages to quickly fix limbs or joints. The splint can be transparent by X-ray. The preservation of amputated limbs during transport is of great significance to the success of replantation. Nursing staff need to convert amputated limbs from warm ischemia to cold ischemia as soon as possible. At present, the method in our hospital is to store the severed limbs in a dry incubator at about 4°C for isolation, which can effectively reduce the reproduction and growth of bacteria that pollute the limbs and reduce the incidence of infection after surgery. Avoid direct contact of limbs with ice cubes. Do not immerse limbs in any liquid, including normal saline; otherwise, if the time is too long, the tissue will swell, and the amputated limb will lose the possibility of replantation.

However, there are still some shortcomings in this study, with the hope of subsequent improvement: (1) this study is a retrospective study, with a low level of evidence, and prospective studies can be designed in the later period; (2) the quantity of experimental patients is small, and the evaluation indicators are relatively few. We will continue to follow up with these patients to record their limb function scores.

## 5. Conclusion

Standardized emergency specialist nursing measures combined with green channel mode can effectively shorten the preoperative examination time and help improve the success rate of amputated limb replantation surgery.

## Figures and Tables

**Figure 1:** Special insulation box for an amputated limb.

**Table 1:** The preoperative examination time and replantation success rate in the control group and experimental group.

	Control group	Experimental group	*P* value
Age	3.8 ± 0.7	0.8 ± 0.7	.954
Preoperative examination time	15.1 ± 3.1	23.2 ± 1.5	*0.0001*
Replantation success rate	72.2%	81.8%	*<0.05*

## Data Availability

The data used to support this study are available from the corresponding author upon request.

## References

[1] Parashar A., Sharma R., Kaladagi R., Nair S., Shetty H. (2020). Major upper limb replantation: an account of patient tenacity. *Plastic and Reconstructive Surgery. Global Open*.

[2] Hui Z., Bin Z., Jie C. (2021). The application of the emergency green channel integrated management strategy in intravenous thrombolytic therapy for AIS. *American Journal of Translational Research*.

[3] Hohenberger G. M., Konstantiniuk P., Cambiaso-Daniel J. (2020). The mangled extremity severity score fails to be a good predictor for secondary limb amputation after trauma with vascular injury in Central Europe. *World Journal of Surgery*.

[4] Siracuse J. J., Farber A., Cheng T. W., Jones D. W., Kalesan B. (2020). Lower extremity vascular injuries caused by firearms have a higher risk of amputation and death compared with non-firearm penetrating trauma. *Journal of Vascular Surgery*.

[5] van Dongen T. T., Huizinga E. P., de Kruijff L. G. (2017). Amputation: not a failure for severe lower extremity combat injury. *Injury*.

[6] Jang Y. S., Lee B. H., Park H. S. (2017). Lower amputation rate after fasciotomy by straight midline incision technique for a 22,900-V electrical injury to the upper extremities. *Injury*.

[7] Bhatnagar V., Richard E., Melcer T., Walker J., Galarneau M. (2019). Retrospective study of cardiovascular disease risk factors among a cohort of combat veterans with lower limb amputation. *Vascular Health and Risk Management*.

[8] Schechtman David W., Walters Thomas J., Kauvar David S. (2021). Utility of the mangled extremity severity score in predicting amputation in military lower extremity arterial injury. *Annals of Vascular Surgery*.

[9] Katiyar A. K., Agarwal H., Priyadarshini P. (2020). Primary vs delayed primary closure in patients undergoing lower limb amputation following trauma: a randomised control study. *International Wound Journal*.

[10] Tillmann B. W., Guttman M. P., Nathens A. B., de Mestral C., Kayssi A., Haas B. (2021). The timing of amputation of mangled lower extremities does not predict post-injury outcomes and mortality: a retrospective analysis from the ACS TQIP database. *Journal of Trauma and Acute Care Surgery*.

[11] Resnik L., Borgia M., Silver B., Cancio J. (2017). Systematic review of measures of impairment and activity limitation for persons with upper limb trauma and amputation. *Archives of Physical Medicine and Rehabilitation*.

[12] Krueger C. A., Rivera J. C., Tennent D. J., Sheean A. J., Stinner D. J., Wenke J. C. (2015). Late amputation may not reduce complications or improve mental health in combat-related, lower extremity limb salvage patients. *Injury*.

[13] Nayar S. K., Alcock H. M., Edwards D. S. (2022). Primary amputation versus limb salvage in upper limb major trauma: a systematic review. *European Journal of Orthopaedic Surgery and Traumatology*.

[14] van den Akker L. E., Holla J. F., Dadema T. (2020). Determinants of physical activity in wheelchair users with spinal cord injury or lower limb amputation: perspectives of rehabilitation professionals and wheelchair users. *Disability and Rehabilitation*.

[15] Jain A., Glass G. E., Ahmadi H. (2013). Delayed amputation following trauma increases residual lower limb infection. *Journal of Plastic, Reconstructive & Aesthetic Surgery*.

[16] Nawijn F., Westenberg R. F., Langhammer C. G., Chen N. C., Eberlin K. R. (2020). Factors associated with primary and secondary amputation following limb-threatening upper extremity trauma. *Plastic and Reconstructive Surgery*.

[17] Polcz J. E., White J. M., Ronaldi A. E. (2021). Temporary intravascular shunt use improves early limb salvage after extremity vascular injury. *Journal of Vascular Surgery*.

